The article "De novo Cancers Following Liver Transplantation: A Single Center Experience in China" was retracted in 2019. Reasons: lack of ethics approval or compliance; missing or withdrawn patient consent; ethical violations by an author.

# *De novo* Cancers Following Liver Transplantation: A Single Center Experience in China

**DOI:** 10.1371/journal.pone.0085651

**Published:** 2014-01-24

**Authors:** Songfeng Yu, Feng Gao, Jun Yu, Sheng Yan, Jian Wu, Min Zhang, Weilin Wang, Shusen Zheng

**Affiliations:** 1 Division of Hepatobiliary and Pancreatic Surgery, Department of Surgery, First Affiliated Hospital, School of Medicine, Zhejiang University, Hangzhou, China; 2 Key Laboratory of Combined Multi-Organ Transplantation, Ministry of Public Health, First Affiliated Hospital, School of Medicine, Zhejiang University, Hangzhou, China; 3 Key Laboratory of Organ Transplantation, Zhejiang Province, Hangzhou, China; SRI International, United States of America

## Abstract

**Background:**

*De novo* cancers are a growing problem that has become one of the leading causes of late mortality after liver transplantation. The incidences and risk factors varied among literatures and fewer concerned the Eastern population.

**Aims:**

The aim of this study was to examine the incidence and clinical features of *de novo* cancers after liver transplantation in a single Chinese center.

**Methods:**

569 patients who received liver transplantation and survived for more than 3 months in a single Chinese center were retrospectively reviewed.

**Results:**

A total of 18 *de novo* cancers were diagnosed in 17 recipients (13 male and 4 female) after a mean of 41±26 months, with an overall incidence of 3.2%, which was lower than that in Western people. Of these, 8 (3.32%) cases were from 241 recipients with malignant liver diseases before transplant, while 10 (3.05%) cases were from 328 recipients with benign diseases. The incidence rates were comparable, p = 0.86. Furthermore, 2 cases developed in 1 year, 5 cases in 3 years and 11 cases over 3 years. The most frequent cancers developed after liver transplantation were similar to those in the general Chinese population but had much higher incidence rates.

**Conclusions:**

Liver transplant recipients were at increased risk for developing *de novo* cancers. The incidence rates and pattern of *de novo* cancers in Chinese population are different from Western people due to racial and social factors. Pre-transplant malignant condition had no relationship to *de novo* cancer. Exact risk factors need further studies.

## Introduction

Liver transplantation (LTx) is the sole curative option for patients with end-stage liver diseases. With the improvement of immunosuppression and other refinements in the management of patients after LTx, graft and patient survivals have markedly increased. Many centers have reported the graft and patient survival rates over 90% for 1 year and close to 80% for 5 years [1]. Therefore, long-term complications after LTx become more important. Among these, development of cancers (recurrence or *de novo*) after LTx is a growing problem leading to an increased late mortality with a functioning graft [2].

Patients who underwent LTx for liver malignant diseases such as hepatocellular carcinoma (HCC) have a potential risk of disease recurrence post transplantation. Up to date, intensive studies have focused on tumor recurrence towards optimizing the candidate criteria and tumor surveillance in such population [3]. On the other hand, studies on *de novo* cancers after LTx in patients without pre-existing malignancies before LTx are rising. In recent years, several reports have clearly shown increased incidences of various types of *de novo* cancers following LTx [4]–[10]. Though mechanisms for the posttransplant *de novo* cancer remain unclear, the etiology is believed to be multifactorial. Immunosuppression is proposed to play a major role in the oncogenesis, both through impaired immunosurveillance and through direct carcinogenic effect of agents [11]. Other potential factors such as viral infection, longer survival, oncogene adoptive transfer from donors, age, gender et al could also be involved [12], [13].

The reported incidence of developing *de novo* cancers ranged from 2.3 to 26%, depending on the demographics of the recipients, length of follow-up, and the era in which transplantations were performed [13], [14]. The most common *de novo* cancers reported in literatures were skin cancers followed by posttransplantation lymphoproliferative disorder (PTLD) [13]. However, most of the studies were performed in Western countries. As the epidemiology of various cancers varies markedly in different geographic eras and ethnic populations, for example skin cancer is relatively rare in Eastern people, we thus reviewed our series for the incidence and pattern of *de novo* cancers that might develop after LTx in Chinese population.

## Materials and Methods

From a maintained database, we retrospectively reviewed all the patients who underwent orthotopic liver transplantation between January 2005 and December 2011 at the first affiliated hospital, school of medicine, Zhejiang university. Patients who survived at least 3 months after transplantation were enrolled in this study. Those who received combined organ transplantation or had previously undergone transplantation were excluded. Clinical data from patients who developed *de novo* cancers post transplantation were collected including primary diagnosis, immunosuppression regimen, type of cancer, elapse time from LTx to diagnosis of cancer, and patient survival. Ethical approval was obtained from the Committee of Ethics in Biomedical Research of Zhejiang University and conformed to the ethical guidelines of the 1975 Declaration of Helsinki. Written informed consent was obtained from all participants.

The primary immunosuppression regimen consisted a triple regimen of tacrolimus (FK506) in combination with mycophenolate mofetil (MMF) and prednisolone for patients with benign end stage liver diseases. The dose of prednisolone was tapered to 5 mg daily 6 weeks post transplantation and was withdrawn after 3 months. Patients underwent LTx for HCC received an induce therapy with Basiliximab and steroid-free regimen. The target blood trough level of FK506 was 7–10 ng/ml for the first post-operative month and aimed at 5–7 ng/ml thereafter. MMF was discontinued when drug specific complications occurred. For some patients, FK 506 monotherapy was achieved after long time stable survival. All the patients were followed up weekly until stable, and then monthly, including regular monitoring biochemical parameters and drug concentration. Image surveillance was also conducted with ultrasound every month and computed tomography for abdomen and chest every half a year.

Data were express as mean value and standard deviation and analyzed with the statistical software package SPSS 15.0. Statistical analyses were carried out using the chi-square test (noncontinuous variables), Kaplan-Meier method with log-rank test (patient survival), Student's t-test (continuous variables with normal distribution) and the Mann–Whitney U-test (continuous variables with nonparametric distribution). A p value<0.05 was considered statistically significant.

## Results

### Risk factor for *de novo* cancers after LTx

During the study period, a total of 569 patients underwent LTx at our center and survived at least 3 months after transplantation were enrolled for the retrospective study. Out of the 569 patients (492 male and 77 female, mean age 47.4±9.7 years), a total of 18 *de novo* cancers were diagnosed in 17 patients (13 male and 4 female) after a mean of 41±26 months (8 to 85 months), with an overall incidence of 3.2%. Results from our series showed that female recipients were more likely to develop *de novo* cancer (4/77 vs. 13/492). Figure 1A shows the risk of *de novo* cancer after LTx were significantly higher in female than male (p = 0.015).

**Figure 1:** Risk of *de novo* cancer after liver transplantation in patients survived more than 3 months after transplantation according to their (A) ages, (B) genders and (C) pre-transplant tumor status.

In general population, young adults have lower risk of tumor, and this risk increases with age. According to the patient age at transplantation, we divided the patients of our series into three groups: <40, 40–50 and >50 years. Although there was no significant difference for the risks of *de novo* cancer after LTx in three groups (p>0.05), patients younger than 40 years seemed to have lower risk during late period after LTx than the elder patients (Figure 1B).

To determine whether pre-transplant malignant conditions could increase the incidence of *de novo* cancer after transplantation, 569 patients were divided into two groups. 241 patients were primarily diagnosed with malignant liver disease before LTx (malignant group), while 328 patients underwent LTx for benign end stage liver disease (non-malignant group). All the patients had no evidence of extrahepatic malignancies before LTx. The patients' details and *de novo* cancer incidences for the two groups are listed in Table 1. There were differences in the patient ages and sex compositions between the two groups, with younger individuals and more males in the malignant group. For the types of LTx, patients in the malignant group underwent more cadaveric liver transplantation and less living donor liver transplantation than those in non-malignant group (90.9% and 9.1% vs. 72.6% and 27.4%, respectively). There were also significant differences in the follow-up time and patient survival rates between the two groups. Patients in the non-malignant group had longer follow-up time (52.7±26.8 months vs. 37.1±27.9 months) than those in the malignant group. There were 8 cases of *de novo* cancer developed in the malignant group and 10 cases in the non-malignant group. The incidence rates were comparable between the two groups (3.32% vs. 3.05%, p = 0.86) with an odds ratio 0.92. Hazard plots showed pre-transplant tumor status had no influence on the risks of *de novo* cancer after LTx (Figure 1C). There was also no difference for the elapse time from LTx to *de novo* cancer between the two groups (44.0±24.9 months vs. 44.5±29.0 months, p = 0.97).

**Table 1:** Clinical details and *de novo* cancer incidences in recipients who underwent LTx for primary diagnosis of malignant and non-malignant disease.

	Malignant group	Non-malignant group	P value
No. of patients	241	328	
Gender			
Male	219	273	0.009
Female	22	55	
Age (yr)	45.5±9.9	49.9±8.9	<0.001
Type of LTx			
Cadaveric	201 (90.9%)	238 (72.6%)	0.002
LDLT	40 (9.1%)	90 (27.4%)	
Follow-up (mo)	37.1±27.9	52.7±26.8	<0.001
No. of *de novo* cancers	8 (3.32%)	10 (3.05%)	0.86Δ
Elapse time from LTx to cancer (mo)	44.0±24.9	44.5±29.0	0.97

**LTx**, liver transplantation; **LDLT**, living donor liver transplantation.

Follow up time and age are expressed as the mean±SD.

Δ Odds Ratio: 0.92.

### Prevalence of *de novo* cancers after LTx

Among the 18 *de novo* cancers, twelve types were identified. The most developed *de novo* cancer was PTLD (n = 3), followed by cancers in liver, stomach, lung, and cervix with 2 cases of each. Other less frequent cancers identified were pancreatic cancer, renal cancer, acute myeloid leukemia (M2a), myelodysplastic syndromes-refractory anemia with excess blasts (MDS-RAEB) and nasopharyngeal cancer. In addition, one patient presented a huge mass in the abdominal wall after a long-tem incision infection due to anastomotic fistula of cholangiojejunostomy. Biopsy only showed poorly differentiated adenocarcinoma infiltrating in the fibrous tissue of abdominal wall but did not identify its origin. She died 6 months after diagnosis lacking effective treatment. The patient who developed nasopharyngeal cancer also developed lung cancer 2 years later and died from complications of lung cancer. Most of the patients received one or two aggressive treatments including operation, chemotherapy, and radiotherapy. Over a mean follow-up period of 21.4±21.0 months (range 1 to 89) after diagnosis of *de novo* cancers, 8 patients (47.1%) died. The causes of death were all related to the *de novo* cancers. The median survival time was 14 months. The demographic and clinical features of these patients are shown in Table 2.

**Table 2:** Demographic and clinical features of the patients with *de novo* malignancy.

Patient No.	Sex/Age	Primary diagnosis	Type of LTx	Immuno-suppression	*De novo* malignancy	Time of occur (m)*	Treatment	Follow-up (m)#	Status
1	M/50	HCC	Cadaveric	FK+MMF	PTLD	24	CTx+RTx	4	Dead
2	M/43	HBV LC	Cadaveric	FK	PTLD	43	None	1	Dead
3	M/49	HBV LC	Cadaveric	FK	PTLD	12	OP+CTx	89	Alive
4	F/60	HCC	Cadaveric	FK	MDS-RAEB	37	None	3	Dead
5	M/48	HCC	LDLT	FK	AML-M2a	27	CTx	11	Dead
6	M/54	HBV LC	Cadaveric	FK+MMF	HCC	42	TACE	17	Dead
7	M/36	HBV LC	LDLT	FK+MMF	HCC	23	RFA+RTx	10	Dead
8	M/48	HCC	Cadaveric	FK	Pancreatic cancer	85	CTx	11	Alive
9	M/55	HBV LC	Cadaveric	FK	Gastric cancer	73	OP+CTx	20	Alive
10	M/58	Alcoholic LC	Cadaveric	FK+MMF	Gastric cancer	40	OP	24	Alive
11	M/52	HCC	Cadaveric	FK	Colon cancer	22	OP	24	Alive
12	M/49	HBV LC	Cadaveric	FK	Renal cancer	84	OP	9	Alive
13	F/40	HCC	Cadaveric	FK	Lung cancer	13	OP	40	Alive
14	M/52	HCC	Cadaveric	FK	Nasopharyngeal cancer	63	RTx	32	
					Lung cancer	85	CTx	10	Dead
15	F/47	HBV LC	Cadaveric	FK	Cervix cancer	56	OP	37	Alive
16	F/49	HBV LC	Cadaveric	FK	Cervix cancer	59	OP	38	Alive
17	F/50	Cholelithiasis	Cadaveric	FK+MMF	Adenocarcinoma in abdominal wall	8	None	6	Dead

**HCC**, hepatocellular carcinoma; **HBV**, hepatitis B virus; **LC**, liver cirrhosis; **LDLT**, living donor liver transplantation; **FK,** tacrulimus; **MMF**, mycophenolate mofetil; **PTLD**, post-transplant lymphoproliferative disorders; **MDS-RAEB**, Myelodysplastic syndromes-refractory anemia with excess blasts; **AML**, acute myeloid leukemia; **CTx**, chemotherapy; **RTx**, radiotherapy; **OP**, operation; **TACE**, transcatheter arterial chemoembolization; **RFA**, radiofrequency ablation;

* Time period from liver transplantation to *de novo* cancer;

# time period from the diagnosis of *de novo* cancer to last follow-up.

According to the report of cancer incidences in China from 2003 to 2007 [15], the most frequent *de novo* cancers in the LTx recipient were similar to the most cancers developed in the general Chinese population. Furthermore, as summarized in Table 3, the incidence rates of either overall or most common cancers were much higher in LTx recipients, suggesting a higher relative risk of cancers following LTx than in the general population.

**Table 3:** Incidence rates of the common cancers in the Chinese general population and liver transplantation patients (per 10^5^ persons).

	Over all		Male		Female	
	General population#	LTx recipients	General population#	LTx recipients	General population#	LTx recipients
Overall	265.93	3163.44	293.99	2642.23	237.19	6493.51
Lymphoma (PTLD*)	6.54	527.24	7.53	609.75	5.48	-
Lung cancer	48.90	351.49	64.59	203.25	32.83	1298.70
Gastric cancer	33.14	351.49	44.36	406.50	21.65	-
HCC	26.68	351.49	39.42	406.50	13.63	-
Cervix cancer	-	-	-	-	9.62	2597.40

**LTx,** liver transplantation; **HCC,** hepatocellular carcinoma; **PTLD,** post transplantation lymphoproliferative disorders.

* Disease name for liver transplantation patients.

# Reported incidence in Chinese population between 2003–2007.

### *De novo* cancers increase late mortality in LTx recipients

Further analysis for the elapse time from LTx to *de novo* cancer showed 2 cases developed in 1 year, 5 cases in 3 years and 11 cases over 3 years, indicating the incidence of *de novo* cancer increased as the patient survival accrued after LTx (Figure 2). To determine the role of *de novo* cancers in the causes of patient death after LTx, we excluded those who died of tumor recurrence, as which has been considered a major cause of death after LTx for patient with malignant liver disease. Kaplan-Meier survival analysis showed that patients with *de novo* cancers had significantly lower survival than the control patients after excluding those who died of tumor recurrence (p = 0.009, Figure 3). This suggests that compared with non-tumor factors *de novo* cancer has contributed more to the patient later mortality after LTx.

**Figure 2:** The number of *de novo* cancer cases developed in the different follow-up years after liver transplantation.

**Figure 3:** Kaaplan-Meier survival analysis for patients with and without *de novo* cancer after liver transplantation. Patients without *de novo* cancer who died of tumor recurrence were excluded from comparison.

## Discussion

In our series involving 569 patients of LTx over a 6 years period, *de novo* cancers were developed in 3.2% of patients at a mean interval of 41 months from the time of LTx. This incidence was among the lowest reported rate from the previous literatures. The highest incidence of posttransplant cancer was reported by a Spanish group, a rate of 26% (49 cases) in a cohort of 187 LTx recipients [16]. Baccarani et al from Italy reported an incidence of 10.3% of *de novo* malignancies in a series of 417 LTx patients survived for more than 30 days and without a previous diagnosis of cancer [4]. A larger series from a single center study by Jain et al in USA showed 6% of 1,127 LTx patients developed *de novo* cancers with a mean follow-up period of 34.1 months [8]. More recently, a 20-year experience from a single European center reported 71 (9.5%) out of 742 patients developed *de novo* neoplasm at a mean time period of 5 years after LTx [5]. Another similar single center study in USA reported the incidence was 13.7% in 534 recipients, which was significantly higher than that in matched population [9]. Results were similar in multicentric studies. Ettorre et al collected 1675 LTx recipients in six Italian transplantation centers and showed a total of 98 patients (5.9%) were diagnosed with *de novo* cancers after 5.2 years [10]. One cohort study in Australia using population-based liver (n = 1926) and cardiothoracic (n = 2718) registries showed the risk of any cancer in liver and cardiothoracic recipients was significantly elevated compared to the general population [17]. Another national wide study of the OPTN/UNOS database showed that in a cohort of 43,196 adult liver recipients 1,923 developed *de novo* malignancy representing an incidence of 4.46% [18]. Only Park et al [6] and Saigal et al [19] reported the incidence rates less than 3%, which were 2.3% and 2.6%, respectively. The possible explanations for the discrepancies in the reported incidence rates may include differences in the size of studied population, the length of follow-up and the era in which LTx was performed. However it is noteworthy that most of those studies were performed in Western populations. Although Saigal et al reported a lower incidence rate, they did not include lymphoid tumors that were more common in other studies, suggesting the real incidence might higher. Only two studies were conducted in Eastern population to date. Park et al reported that out of 1,952 Korean adult LTx recipients, 44 patients (2.3%) were diagnosed with *de novo* cancer at a mean period of 41±29 months. In another Japanese population-based study, Kaneko et al showed 27 *de novo* malignancies were diagnosed in 26 out of 360 adult living donor liver transplantation recipients during an even longer follow-up period [20]. In the present study, the incidence of *de novo* cancers was similar to the Korean group at a comparable length of follow-up period, but lower than that in Western populations. Therefore we suggested that the incidence rates of *de novo* cancers after LTx were different between Eastern and Western people, with more prevalence in the latter. One possible explanation might be that the somatotype of people in Eastern was much smaller than in Western, thus requiring lower dose of immunosuppressants such as calcineurin inhibitor that was considered to be carcinogenic. However the exact mechanism need further study.

It has been clear that the risk factor of *de novo* cancer is multifactorial. Recent studies have suggested that immunosuppression, age and other factors specific for different types of cancer were involved in the development of *de novo* cancers after LTx. First, the intensity of life-long immunosuppressive treatment could be the major reason for this serious complication [21]. Because exogenous immunosuppression is believed to suppress the host defense system including T cells, macrophages and natural killer cells, which normally provide surveillance and protection from oncogenic virus infection and even, destroy tumor cells [22]. Some studies have shown many immunosuppressive agents were related to a higher incidence of *de novo* cancer, for instance, azathioprine and cyclosporine to cutaneous neoplasia [23], tacrolimus to haematological malignancies [21]. Furthermore, patients receiving tacrolimus had a higher risk of neoplasia than those receiving cyclosporine [16], [24]. On the other hand, withdrawal of immunosuppressive drug could result in regression of PTLD in many cases [25]. In our series, most patients received tacrolimus based therapy and only few shifted to cyclosporine. And all the patients developed *de novo* cancer received tacrolimus based regimen. Thus we could not figure out the drug specific relevancy for the *de novo* cancers. Age is another important risk factor. Reports from different centers have found that patients greater than 40 years old [26], 51 years old [27] and 60 years old [28] at time of LTx were an independent risk factor for *de novo* cancer. However, another single center trial reported by Jonas et al found no difference in ages between transplant recipients with and without *de novo* cancers [29]. Results from the present study showed that there was no statistical difference for the risk of *de novo* cancer according to the patient age at LTx (<40 years, 40–50 years and >50 years), p>0.05. However, as further follow-up accrued, recipients who were younger than 40 years presented a significant lower risk compared with the elder recipients (Figure 1B). Gender is not determined as a risk factor of *de novo* cancer. Some studies did not find significant difference between males and female in developing *de novo* cancers [29], [30]. But some did, at least in univariate analysis [16]. Our data showed a significantly increased risk of *de novo* cancer in female recipients after LTx, suggesting a gender involved risk factor. The low incidence and great uneven distribution of numbers between male and female may be one of the causes. Thus more case numbers in female group are needed for further study.

Given the role of immune system in tumor surveillance, evidence is accumulating that patients with premalignant conditions before LTx could have higher risk for developing cancers in the setting of immunosuppression, for example, the relationship between Barrett's oesophagus and oesophageal cancer, colonic polyp and colon cancer, Budd-Chiari syndrome and acute leukemia [31]. It is also clear that patients underwent LTx for malignant liver diseases have a high risk of tumor recurrence. However, no evidence has been clarified whether malignant conditions before LTx could be a risk factor for developing *de novo* cancers after LTx. Our results indicated that the incidence rates were comparable between patients who had malignant liver diseases at time of transplant and those with benign diseases. This was in accordance with the observations form Herrero et al showing HCC was not a risk factor for the development of *de novo* cancer after LTx [16]. Indeed, some specific factors have been suggested for certain cancer types. For example, PTLD can be considered an opportunistic infectious complication usually involving the Epstein-Barr virus [32]. HCC is associated with hepatitis B virus (HBV) recurrence after LTx [33]. In our series, all the patients developed PTLD were detected Epstein-Barr virus positive after LTx, and the two patients with *de novo* HCC had HBV recurrence before developing HCC, thus supporting the previous findings.

From the previous studies, the most common *de novo* cancer after organ transplantation was skin cancer followed by PTLD in Western populations [13]. However, unlike Western countries, no skin cancer was diagnosed among our series. Similar finding was also reported in a study from Taiwan, which reviewed 560 renal transplant recipients for the pattern of cancer occurring after transplantation [34]. Another larger series report from a liver transplant center in Korea also noted that the incidence of skin cancer was relatively low among Korean LTx recipients (only 2 skin cancer in a total of 44 *de novo* cancers after LTx) [6]. The Japanese study also showed that colorectal cancer was the most commonly detected malignancy after living donor liver transplantation [20]. Moreover, the most common *de novo* cancers in our series were PTLD followed by lung cancer, gastric cancer and HCC. According to the common cancer incidence in Chinese general population, the top frequent cancers are lung cancer, gastric cancer, colorectal cancer and liver cancer [15]. The spectrum of cancers between LTx recipients and the general population was almost comparable. While based on our results, the relative risks of overall and individual *de novo* cancer were significantly higher in LTx recipients compared with in the Chinese general population (Table 3). Taken together, our results together with others, suggested that patterns of *de novo* cancer after organ transplantation might differ between Western and Eastern countries. Racial and social factors, including endemic environment could be the underlying explanation.

Recipients of organ transplantation are subjected to lifelong immunosuppression. Thus an increased incidence of developing cancer is expected in recipients with longer follow-up. The longer transplant recipients survive, the greater the risk of cancer accumulates. This was supported by the results in our series. We noted, as expected, that the number of *de novo* cancers increased as further follow-up accrued. Moreover, though receiving aggressive treatments after diagnosis, poor survival of those patients with *de novo* cancers was noted in our series. All the patients who died after the diagnosis had a direct relationship with the *de novo* cancers. Indeed, the causes of patient later death after LTx are multifactorial including chronic rejection, primary disease recurrence and others. Recent studies have currently considered *de novo* cancer as the second leading cause of death following cardiovascular complications [2], [13]. It has been clear that tumor recurrence is the major cause of death after LTx for recipients of malignant liver disease [35]. However, after excluding the patients who died of tumor recurrence, our single center study showed that the survival of patients with *de novo* cancers was significantly lower than those without *de novo* cancers, suggesting that compared with non-tumor factors *de novo* cancer has contributed more to the later mortality after LTx in Chinese population.

## Conclusion

Our findings suggested that liver transplant recipients were at increased risk for developing *de novo* cancers after LTx. The incidence rates and spectrum of *de novo* cancers in Chinese population were different from Western people due to racial and social factors. Gender and age might be the risk factors but pre-transplant malignant condition had no relationship to *de novo* cancer. However, further studies were still needed. The increased prevalence of *de novo* cancer during accrued patient survival was the main cause of patient later mortality after LTx.

## References

[1] MerionRM (2010) Current status and future of liver transplantation. Semin Liver Dis 30: 411–421.2096038010.1055/s-0030-1267541

[2] FungJJ, JainA, KwakEJ, KusneS, DvorchikI, et al (2001) De novo malignancies after liver transplantation: a major cause of late death. Liver Transpl 7: S109–118.1168978310.1053/jlts.2001.28645

[3] SamuelD, ColomboM, El-SeragH, SobeskyR, HeatonN (2011) Toward optimizing the indications for orthotopic liver transplantation in hepatocellular carcinoma. Liver Transpl 17 Suppl 2: S6–13.2185891210.1002/lt.22423

[4] BaccaraniU, PiselliP, SerrainoD, AdaniGL, LorenzinD, et al (2010) Comparison of de novo tumours after liver transplantation with incidence rates from Italian cancer registries. Dig Liver Dis 42: 55–60.1949779710.1016/j.dld.2009.04.017

[5] SapisochinG, BilbaoI, DopazoC, CastellsL, LazaroJL, et al (2011) Evolution and management of de novo neoplasm post-liver transplantation: a 20-year experience from a single European centre. Hepatol Int 5: 707–715.2148410710.1007/s12072-010-9231-1PMC3090551

[6] ParkHW, HwangS, AhnCS, KimKH, MoonDB, et al (2012) De novo malignancies after liver transplantation: incidence comparison with the Korean cancer registry. Transplant Proc 44: 802–805.2248350010.1016/j.transproceed.2012.01.027

[7] YaoFY, GautamM, PaleseC, RebresR, TerraultN, et al (2006) De novo malignancies following liver transplantation: a case-control study with long-term follow-up. Clin Transplant 20: 617–623.1696848810.1111/j.1399-0012.2006.00527.xPMC4050657

[8] JainA, FiazO, SheikhB, SharmaR, SafadjouS, et al (2009) Recurrent nonhepatic and de novo malignancies after liver transplantation. Transplantation 88: 706–710.1974146910.1097/TP.0b013e3181b3918e

[9] ChatrathH, BermanK, VuppalanchiR, SlavenJ, KwoP, et al (2013) De novo malignancy post-liver transplantation: a single center, population controlled study. Clin Transplant 27: 582–590.2380880010.1111/ctr.12171PMC3740024

[10] EttorreGM, PiselliP, GalatiotoL, RendinaM, NudoF, et al (2013) De novo malignancies following liver transplantation: results from a multicentric study in central and southern Italy, 1990–2008. Transplant Proc 45: 2729–2732.2403403410.1016/j.transproceed.2013.07.050

[11] DantalJ, SoulillouJP (2005) Immunosuppressive drugs and the risk of cancer after organ transplantation. N Engl J Med 352: 1371–1373.1580023410.1056/NEJMe058018

[12] PopovZ, IvanovskiO, KolevskiP, StankovO, PetrovskiD, et al (2007) De novo malignancies after renal transplantation–a single-center experience in the Balkans. Transplant Proc 39: 2589–2591.1795418410.1016/j.transproceed.2007.08.022

[13] ChakE, SaabS (2010) Risk factors and incidence of de novo malignancy in liver transplant recipients: a systematic review. Liver Int 30: 1247–1258.2060268210.1111/j.1478-3231.2010.02303.x

[14] HerreroJI (2009) De novo malignancies following liver transplantation: impact and recommendations. Liver Transpl 15 Suppl 2: S90–94.1987702510.1002/lt.21898

[15] ChenW, ZhengR, ZhangS (2012) An Analysis of Cancer Incidence in China, 2003–2007. China Cancer 21: 161–170.

[16] HerreroJI, LorenzoM, QuirogaJ, SangroB, PardoF, et al (2005) De Novo neoplasia after liver transplantation: an analysis of risk factors and influence on survival. Liver Transpl 11: 89–97.1569054110.1002/lt.20319

[17] NaR, GrulichAE, MeagherNS, McCaughanGW, KeoghAM, et al (2013) Comparison of de novo cancer incidence in Australian liver, heart and lung transplant recipients. Am J Transplant 13: 174–183.2309478810.1111/j.1600-6143.2012.04302.x

[18] SampaioMS, ChoYW, QaziY, BunnapradistS, HutchinsonIV, et al (2012) Posttransplant malignancies in solid organ adult recipients: an analysis of the U.S. National Transplant Database. Transplantation 94: 990–998.2308555310.1097/TP.0b013e318270bc7b

[19] SaigalS, NorrisS, MuiesanP, RelaM, HeatonN, et al (2002) Evidence of differential risk for posttransplantation malignancy based on pretransplantation cause in patients undergoing liver transplantation. Liver Transpl 8: 482–487.1200434910.1053/jlts.2002.32977

[20] KanekoJ, SugawaraY, TamuraS, AokiT, SakamotoY, et al (2013) De novo malignancies after adult-to-adult living-donor liver transplantation with a malignancy surveillance program: comparison with a Japanese population-based study. Transplantation 95: 1142–1147.2357212810.1097/TP.0b013e318288ca83

[21] BenllochS, BerenguerM, PrietoM, MorenoR, San JuanF, et al (2004) De novo internal neoplasms after liver transplantation: increased risk and aggressive behavior in recent years? Am J Transplant 4: 596–604.1502315210.1111/j.1600-6143.2004.00380.x

[22] PennI (1994) Depressed immunity and the development of cancer. Cancer Detect Prev 18: 241–252.7982234

[23] EuvrardS, KanitakisJ (2006) Skin cancers after liver transplantation: what to do? J Hepatol 44: 27–32.1629090910.1016/j.jhep.2005.10.010

[24] WimmerCD, AngeleMK, SchwarzB, PratschkeS, RentschM, et al (2013) Impact of cyclosporine versus tacrolimus on the incidence of de novo malignancy following liver transplantation: a single center experience with 609 patients. Transpl Int 26: 999–1006.2395210210.1111/tri.12165

[25] StarzlTE, NalesnikMA, PorterKA, HoM, IwatsukiS, et al (1984) Reversibility of lymphomas and lymphoproliferative lesions developing under cyclosporin-steroid therapy. Lancet 1: 583–587.614230410.1016/s0140-6736(84)90994-2PMC2987704

[26] HaagsmaEB, HagensVE, SchaapveldM, van den BergAP, de VriesEG, et al (2001) Increased cancer risk after liver transplantation: a population-based study. J Hepatol 34: 84–91.1121191210.1016/s0168-8278(00)00077-5

[27] XiolX, GuardiolaJ, MenendezS, LamaC, FiguerasJ, et al (2001) Risk factors for development of de novo neoplasia after liver transplantation. Liver Transpl 7: 971–975.1169903310.1053/jlts.2001.28744

[28] HerreroJI, LucenaJF, QuirogaJ, SangroB, PardoF, et al (2003) Liver transplant recipients older than 60 years have lower survival and higher incidence of malignancy. Am J Transplant 3: 1407–1412.1452560210.1046/j.1600-6143.2003.00227.x

[29] JonasS, RayesN, NeumannU, NeuhausR, BechsteinWO, et al (1997) De novo malignancies after liver transplantation using tacrolimus-based protocols or cyclosporine-based quadruple immunosuppression with an interleukin-2 receptor antibody or antithymocyte globulin. Cancer 80: 1141–1150.930571610.1002/(sici)1097-0142(19970915)80:6<1141::aid-cncr18>3.0.co;2-8

[30] KellyDM, EmreS, GuySR, MillerCM, SchwartzME, et al (1998) Liver transplant recipients are not at increased risk for nonlymphoid solid organ tumors. Cancer 83: 1237–1243.9740091

[31] MenachemY, SafadiR, AshurY, IlanY (2003) Malignancy after liver transplantation in patients with premalignant conditions. J Clin Gastroenterol 36: 436–439.1270298910.1097/00004836-200305000-00016

[32] JainA, NalesnikM, ReyesJ, PokharnaR, MazariegosG, et al (2002) Posttransplant lymphoproliferative disorders in liver transplantation: a 20-year experience. Ann Surg 236: 429–436; discussion 436–427.1236867110.1097/00000658-200210000-00005PMC1422597

[33] FariaLC, GigouM, Roque-AfonsoAM, SebaghM, RocheB, et al (2008) Hepatocellular carcinoma is associated with an increased risk of hepatitis B virus recurrence after liver transplantation. Gastroenterology 134: 1890–1899; quiz 2155.1842426910.1053/j.gastro.2008.02.064

[34] ChiangYJ, ChenCH, WuCT, ChuSH, ChenY, et al (2004) De novo cancer occurrence after renal transplantation: a medical center experience in Taiwan. Transplant Proc 36: 2150–2151.1551878010.1016/j.transproceed.2004.08.013

[35] ZhengSS, XuX, WuJ, ChenJ, WangWL, et al (2008) Liver transplantation for hepatocellular carcinoma: Hangzhou experiences. Transplantation 85: 1726–1732.1858046310.1097/TP.0b013e31816b67e4

